The article "Clinical Efficacy of Yiqi Yangyin Decoction Combined with Docetaxel on Advanced Ovarian Cancer and the Effect on the Levels of Serum Markers VEGF, HE4, and CA125" was retracted in 2023. Reasons: signs of a paper mill; suspected computer-generated content; unreliable results or conclusions; lack of ethics approval or compliance.

# Clinical Efficacy of Yiqi Yangyin Decoction Combined with Docetaxel on Advanced Ovarian Cancer and the Effect on the Levels of Serum Markers VEGF, HE4, and CA125

**DOI:** 10.1155/2022/8401202

**Published:** 2022-03-23

**Authors:** Ning Wang, Fengying Xiao, Hua Shao, Shuai Shi, Yanling Zhou

**Affiliations:** ^1^Department of Clinical Laboratory, Jiaozhou Central Hospital, Qingdao 266300, China; ^2^Operation Room, Jiyang People's Hospital, Jinan 251400, China; ^3^Radiophysics Department, The Affiliated Qingdao Central Hospital of Qingdao University, The Second Affiliated Hospital of Medical College of Qingdao University, Qingdao 266042, Shandong, China; ^4^Department of Rehabilitation Medicine, Qingdao Eighth People's Hospital, Qingdao 266000, China; ^5^Department of Obstetrics, Yantaishan Hospital, Yantai 264000, China

## Abstract

**Objective:**

The study is designed to investigate the therapeutic effect of Yiqi Yangyin Decoction combined with docetaxel on advanced ovarian cancer (OC) patients and the effects on serum markers VEGF, HE4, and CA125.

**Methods:**

92 patients with advanced OC were grouped into the study group and control group. The control group was given the treatment of basic chemotherapy combined with docetaxel. The study group was added the treatment of Yiqi Yangyin Decoction on the basis of the control group. The short-term efficacy, adverse reactions, tumor markers, quality of life, 3-year survival, and T cell subsets of the two groups were observed.

**Results:**

Compared to the control group, the study group's incidence of adverse reactions was lower. VEGF, HE4, and CA125 in the study group were decreased more obviously. The levels of CD3^+^, CD4^+^, and CD4^+^/CD8^+^ were sharply higher in the study group, while CD8^+^ was notably reduced. After treatment, the scores of physical health, social function, and mental health in the study group were notably higher than those in the control group. Compared with the control group, the 3-year survival rate of the study group was notably higher, and the therapeutic effect of the study group was obviously better.

**Conclusion:**

The combination of Yiqi Yangyin Decoction and docetaxel can improve the body immunity and the therapeutic effect of advanced OC, decrease the incidence of adverse reactions, and prolong the survival time, with good safety and effectiveness.

## 1. Introduction

The incidence of ovarian cancer (OC) in China ranks third after cervical cancer and endometrial cancer [1]. Globally, the morbidity and mortality of OC ranks 8th among female malignant tumors, and with an increasing trend [2]. About 25,000 female patients die of OC every year in China, and the mortality rate ranks 10th among female malignant tumors [3]. The diagnosis rate of early OC is low, and many patients have usually advanced to middle and late stages (stage III and IV) at the time of diagnosis. The 5-year survival rate of OC patients is only 10%∼20% [4]. Anemia, emaciation, fatigue, and abnormal ovarian blood flow may occur in advanced OC. Advanced epithelial OC patients have advanced to the advanced stage, and most of them have abdominal metastasis and a large amount of abdominal effusion, which greatly increases the difficulty of clinical treatment and seriously affects the life safety and quality of life of patient [5]. Currently, Western medicine mainly treats OC with surgery, supplemented by chemotherapy and maintenance therapy. However, the postoperative recurrence rate is generally high, while chemotherapy has a great impact on liver and kidney and often accompanied by bone marrow suppression and digestive tract symptoms [6]. Docetaxel is a broad-spectrum antitumor chemotherapy drug, as a new generation of paclitaxel drugs, which acts on paclitaxel resistant cells without cross-drug resistance. Docetaxel has higher solubility and bioavailability in vivo than paclitaxel, and has stronger antitumor activity and less toxic side effects than paclitaxel [7].

The article "Clinical Efficacy of Yiqi Yangyin Decoction Combined with Docetaxel on Advanced Ovarian Cancer and the Effect on the Levels of Serum Markers VEGF, HE4, and CA125" was retracted in 2023. Reasons: signs of a paper mill; suspected computer-generated content; unreliable results or conclusions; lack of ethics approval or compliance.

An increasing number of studies [8–10] have found that traditional Chinese medicines can play an adjuvant role in chemotherapy, which can enhance therapeutic efficacy, reduce adverse drug reactions, and enhance the immunity of OC patients. VEGF, one of the vital tumor vascular growth factors, can increase vascular permeability and promote endothelial cell proliferation and vascular growth [11]. HE4 [12] is a novel tumor marker that exists in human epididymal epithelial cells and is highly expressed in OC serum. CA125 [13, 14] is a tumor marker in serum, and its level is abnormally elevated in cancer tissues. Disease progression and prognosis can be assessed by monitoring its changes.

In our study, 92 patients with advanced OC were selected for adjuvant treatment with Yiqi Yangyin Decoction combined with docetaxel, providing reference for patients to get better treatment.

## 2. Materials and Methods

### 2.1. The General Information

92 patients with advanced OC were selected as the research objects. The patients were grouped into control group and study group. In the control group, patients were 34 to 67 years old, with a median age of 52 years; body weight was 45–73 kg, with a median weight of 61 kg; clinical stage was stage III in 28 patients and stage IV in 18 patients; pathological classification was 21 cases in mucinous cystadenocarcinoma and 25 cases in serous cystadenocarcinoma. In study group, patients were 32 to 65 years old, with a median age of 49 years; body weight was 47–75 kg, with a median weight of 62 kg; clinical stage was stage III in 30 patients and stage IV in 16 patients; pathological classification was mucinous cystadenocarcinoma in 19 cases and serous cystadenocarcinoma in 27 cases. The general data between the two groups had no significant differences (*p* > 0.05).

The article "Clinical Efficacy of Yiqi Yangyin Decoction Combined with Docetaxel on Advanced Ovarian Cancer and the Effect on the Levels of Serum Markers VEGF, HE4, and CA125" was retracted in 2023. Reasons: signs of a paper mill; suspected computer-generated content; unreliable results or conclusions; lack of ethics approval or compliance.

### 2.2. Selection Criteria

Inclusion criteria were as follows: (1) patients were all advanced ovarian epithelial carcinoma, which was confirmed by pathological examination; (2) met the diagnostic criteria in Obstetrics and Gynecology [15]; (3) met the diagnostic criteria for Qi deficiency and blood stasis OC in the TCM Diagnosis and Treatment Guidelines for Malignant Tumors [16]; (4) patients' Karnofsky's performance status (KPS) > 60 [17], with an estimated survival of more than 6 months; (5) patients were 30 to 70 years old; and (6) patients were aware of the content and purpose of the study and have no objection and voluntarily sign the informed consent form.

Exclusion criteria were as follows: (1) patients with other primary tumors, (2) patients with immune system diseases, (3) patients with severe liver or kidney dysfunction, (4) patients who were mentally abnormal and unable to cooperate with the study, and (5) patients who had received radiotherapy and chemotherapy within 3 months before enrollment.

### 2.3. Treatment Methods

The control group was received basic chemotherapy combined with docetaxel. On the first day of chemotherapy, paclitaxel injection (135 mg/m^2^, North China Pharmaceutical Co., Ltd., National drug approval H20084439) was added into sodium chloride injection (0.9%, 250 ml) for intravenous infusion. At the same time, cisplatin injection (60 mg/m^2^, Jiangsu Hausen Pharmaceutical Group Co., Ltd., , National drug approval H20040813) was added into sodium chloride injection (0.9%, 250 ml) for intravenous infusion. Meanwhile, docetaxel injection (70 mg/m^2^, Jiangsu Aosaikang Pharmaceutical Co., LTD., National drug approval H20064301) was added into sodium chloride injection (0.9%, 250 ml) for intravenous infusion. Chemotherapy was given once every three weeks for a total of 6 courses.

Based on the control group, the study group was received adjuvant treatment with Yiqi Yangyin Decoction [18]. The formula was as follows: *Astragalus membranaceus* 35 g, Chinese yam 25 g, Jujube 10 g, *Prunella subtilis* 15 g, *Platycodon grandiflorum* 10 g, Huangjing 15 g, *Fructus ligustris* 20 g, Zedoary turmeric 15 g, Shengdi 20 g, Radix scrophulariae 20 g, Radix Aconitum 20 g. The specific dose can be increased or decreased according to different symptoms of different patients. Patients take one dose of oral medicine twice a day in the morning and twice. There were three weeks for a course of treatment, a total of 6 courses.

The article "Clinical Efficacy of Yiqi Yangyin Decoction Combined with Docetaxel on Advanced Ovarian Cancer and the Effect on the Levels of Serum Markers VEGF, HE4, and CA125" was retracted in 2023. Reasons: signs of a paper mill; suspected computer-generated content; unreliable results or conclusions; lack of ethics approval or compliance.

### 2.4. Observation Indicators and Evaluation Criteria

1. The efficacy of the two groups was evaluated by the response evaluation criteria in solid tumor (RECIST) [19]. Complete response (CR): the lesion was disappeared completely, and the duration was more than one month. Partial response (PR): the product of the tumor maximum and maximum vertical diameters was reduced ≥50%. Stable disease (SD): the product of the tumor maximum and vertical diameters was decreased by <50% or increased by <25%. Progressive disease (PD): the product of tumor maximum and maximum vertical diameters with one or more lesions was increased by ≥ 25%.
2. The fasting venous blood (5 mL) was obtained from the patients in the morning, and stored at −20°C after centrifugation. The levels of VEGF and HE4 were tested by ELISA. The level of carbohydrate antigen 125 (CA125) was detected by automatic analyzer.
3. Patients were followed up for 3 years, and the 3-year cumulative survival was recorded by telephone and consultation.
4. The adverse reactions were compared between the control group and study group, including liver injury, gastrointestinal reactions, bone marrow suppression, cardiotoxicity, neurotoxicity, nausea, and vomiting. The severity was classified as I (mild), II (moderate), and III (severe) from mild to severe.
5. The levels of T lymphocyte subsets were tested by flow cytometry, including CD3^+^, CD8^+^, CD4^+^, and CD4^+^/CD8^+^. The flow cytometry kit should be used and strictly operated according to the instructions of the instrument.
6. Before and after treatment, the quality of life was assessed via the quality of life questionnaire for Chinese cancer patients with chemo bio therapy (QLQ-CCC) [20], including physical health, social function, and mental health.

### 2.5. Statistical Method

SPSS 20.0 was used to analyze the data. The measurement data were represented as $\bar{x}$ ± *s*. The comparisons between the groups were performed by *t*-test. The counting data were represented by the number of cases and the rate (%). *χ*^2^ test was used for comparison between groups. Kaplan–Meier analysis was used to draw the survival curve. When *p* < 0.05, the difference was statistically significant.

## 3. Results

### 3.1. The Short-Term Efficacy between the Two Groups Was Compared

The total effective rate of the study group was 89.13%, which clearly higher than that of the control group (71.74%). There was significant difference of the short-term efficacy between the control group and study group (*p* < 0.05, Table 1).

The article "Clinical Efficacy of Yiqi Yangyin Decoction Combined with Docetaxel on Advanced Ovarian Cancer and the Effect on the Levels of Serum Markers VEGF, HE4, and CA125" was retracted in 2023. Reasons: signs of a paper mill; suspected computer-generated content; unreliable results or conclusions; lack of ethics approval or compliance.

### 3.2. VEGF, HE4, and CA125 Levels between Two Groups Were Compared

VEGF, HE4, and CA125 levels in both groups were significantly declined after treatment. Compared to the control group, the decrease was more pronounced in the study group (Figure 1).

### 3.3. Comparison of T Cell Subsets between the Control Group and Study Group

Compared with before treatment, CD3^+^, CD4^+^, and CD4^+^/CD8^+^ levels in two groups were ascended, while CD8^+^ was declined notably. Compared to the control group, the levels of CD3^+^, CD4^+^, and CD4^+^/CD8^+^ in the study group were higher, and CD8^+^ was lower (*p* < 0.05, Figure 2).

### 3.4. Comparison of Quality of Life between the Control Group and Study Group

Compared with before treatment, the scores of physical health, social function, and mental health in both groups were notably higher, and the increase in study group was more remarkable (*p* < 0.001, Table 2).

### 3.5. Comparison of 3-Year Survival Rate between the Control Group and Study Group

The 3-year survival rate of the study group was 69.57%, which was notably higher than the control group (45.65%) (*p* < 0.05, Figure 3).

### 3.6. Comparison of Adverse Reactions between the Control Group and Study Group

There were no obvious differences in the incidence of liver injury, bone marrow suppression, gastrointestinal reaction, cardiotoxicity, neurotoxicity, nausea, and vomiting between the control group and study group (*p* > 0.05, Table 3).

## 4. Discussion

OC is one of the most common malignant tumors of female reproductive system, which is common in middle-aged and elderly patients. Recently, the new cases of OC are increasing year by year, and the fatality rate is over 60% [4]. Due to the deep anatomical location of OC, it is difficult to diagnose and give clinical intervention in the early stage of the lesion. Cancer cells usually spread to the uterus, adnexa and other organs, resulting in difficult and ineffective treatment. Clinically, paclitaxel combined with platinum drugs is a common and effective chemotherapy for OC. However, with the increase of chemotherapy time, the drug resistance of paclitaxel and carboplatin will reduce the chemotherapy sensitivity of OC patients [21]. In addition, chemotherapy may cause immunosuppression and other complications, affecting the prognosis and life quality. Therefore, on the basis of paclitaxel and platinum drug therapy, the combination of other chemotherapy drugs to improve the effect of tumor intervention and patients' prognosis has become a hot spot of clinical concern. Paclitaxel is an antitumor microangiogenic drug that prevents the mitosis of tumor cell DNA by suppressing the overall aggregation of tubulin. Docetaxel [22] has the same antitumor mechanism as paclitaxel, but its antitumor spectrum is broader than that of paclitaxel.

The article "Clinical Efficacy of Yiqi Yangyin Decoction Combined with Docetaxel on Advanced Ovarian Cancer and the Effect on the Levels of Serum Markers VEGF, HE4, and CA125" was retracted in 2023. Reasons: signs of a paper mill; suspected computer-generated content; unreliable results or conclusions; lack of ethics approval or compliance.

According to traditional Chinese medicine [23], patients are in the state of weakness of Yin and Yang after chemotherapy, easy to form spittoon coagulate, qi stagnation, stasis poison inside knot of the disease. The main effect of Yiqi Yangyin Decoction is to heat and detoxification, nourish qi, and yin. Astmgali Radix can nourish qi and spleen, detumescence, and diuresis. Rehmanniae Radix can clear heat and promote fluid production. Dioscoreae Rhizoma can invigorate spleen and kidney, improve eyesight, and soothe the nerves. *Ligustrum lucidum* Ait can reinforce liver and kidney. Curcumae Rhizoma can regulate qi flowing for relieving pain and resolve hard mass. Scrophulariae Radix can nourish yin and cool blood, clear heat, and remove toxicity. Pseudobulbus Cremastrae seu Pleiones and *Prunella vulgaris* can clear heat, remove toxicity, and reduce swelling, and the combination of the two drugs can accelerate the apoptosis of tumor cells. The combination of these drugs have the function of clearing heat and detoxifying, nourishing qi and Yin, strengthening the body resistance, thus promoting the body to secrete immune factors, with a good effect on adjuvant chemotherapy [24–27]. Our findings displayed that there was no obvious difference in adverse reactions between the two groups. Moreover, Yiqi Yangyin Decoction combined with docetaxel has a significant clinical effect in the treatment of advanced OC and does not cause damage to the liver, gastrointestinal function, and nerve function, so it has a certain safety.

In addition, the distribution of T cell subsets in both groups improved after treatment. The levels of CD3^+^, CD4^+^, CD8^+^, and CD4^+^/CD8^+^ in the study group were sharply better than those in the control group. The study group scored higher in physical health, social function, and mental health, and the 3-year survival rate was higher than the control group. Our results indicated that Yiqi Yangyin Decoction combined with docetaxel can boost the immune function, greatly improve the quality of life, and prolong the survival time. VEGF is a dimer composed of two 24 kD single chains, which can directly act on vascular endothelial cells and increase vascular permeability. VEGF is associated with the occurrence of tumors and can promote the proliferation and differentiation of tumor cells. VEGF is a viral indicator for clinical evaluation of tumor cell proliferation and differentiation and is highly expressed in most tumor tissues [28, 29]. HE4 is a new tumor marker existing in the distal end of renal tubules and epithelium of the reproductive system. HE4 was overexpressed in OC tissues, and its expression level was not affected by the menstrual status of patients. Some studies [30] have shown that the sensitivity of HE4 in the diagnosis of OC is 72.4%. We found that VEGF, HE4, and CA125 levels in the study group were declined more obviously than those of the control group, reflecting that Yiqi Yangyin Decoction combined with docetaxel can reduce the inflammatory response, inhibit tumor growth, and restore the normal level of tumor markers. However, due to the small sample size of the clinical trial in this study, statistical deviation inevitably occurred. Therefore, the sample size and other indicators detected should be increased to improve the study.

The article "Clinical Efficacy of Yiqi Yangyin Decoction Combined with Docetaxel on Advanced Ovarian Cancer and the Effect on the Levels of Serum Markers VEGF, HE4, and CA125" was retracted in 2023. Reasons: signs of a paper mill; suspected computer-generated content; unreliable results or conclusions; lack of ethics approval or compliance.

## 5. Conclusion

To sum up, Yiqi Yangyin Decoction combined with docetaxel can play a good therapeutic effect in advanced OC, reduce the toxic and side effects brought by chemotherapy, reduce the levels of tumor markers, enhance the immune function, and improve the life quality. Therefore, Yiqi Yangyin Decoction combined with docetaxel in the treatment of advanced OC can be an ideal clinical treatment.

## Figures and Tables

**Figure 1:** Comparison of serum VEGF, HE4, and CA125 levels between the two groups. (a) The comparison of serum VEGF levels between the two groups before and after treatment. (b) The comparison of serum HE4 levels between the two groups before and after treatment. (c) The comparison of serum CA125 levels between the two groups before and after treatment.

**Figure 2:** T cell subsets were compared between two groups before and after treatment. (a) Comparison of CD3^+^ level between the two groups. (b) Comparison of CD4^+^ level between the two groups. (c) Comparison of CD8^+^ level between the two groups. (d) Comparison of CD4^+^/CD8^+^ level between the two groups.

**Figure 3:** Comparison of 3-year cumulative survival rate between the two groups.

**Table 1:** Comparison of short-term efficacy between the two groups (*n*, %).

Group	*n*	CR	PR	SD	PD	Total effective rate
Study group	46	25	16	4	1	41 (89.13)
Control group	46	13	20	7	6	33 (71.74)
*χ* ^2^						8.624
*p* value						0.035

**Table 2:** QLQ scores were compared between two groups before and after treatment.

Groups		Physical health	Social function	Mental health
Study group	Before treatment	65.89 ± 6.18	68.30 ± 6.04	61.33 ± 6.03
	After treatment	88.28 ± 4.62	87.35 ± 6.10	85.30 ± 6.10
Control group	Before treatment	67.22 ± 5.96	70.07 ± 6.51	62.26 ± 6.08
	After treatment	76.24 ± 5.90	78.28 ± 6.02	75.28 ± 6.13
*t*		10.890	7.178	7.858
*p* value		0.00	0.00	0.00

**Table 3:** Comparison of adverse reactions between the two groups (*n*, %).

Adverse reactions		Study group (*n* = 46)	Control group (*n* = 46)	*χ* ^2^	*p* value
Liver injury				0.256	>0.05
	0∼I	37	35		
	II∼III	9	11		

Bone marrow suppression				0.214	>0.05
	0∼I	32	34		
	II∼III	14	12		

Gastrointestinal reaction				0.858	>0.05
	0∼I	35	31		
	II∼III	11	15		

Cardiotoxicity				0.522	>0.05
	0∼I	36	33		
	II∼III	10	13		

Neurotoxicity				0.050	>0.05
	0∼I	31	32		
	II∼III	15	14		

Nausea and vomiting				0.425	>0.05
	0∼I	28	31		
	II∼III	18	15		

The article "Clinical Efficacy of Yiqi Yangyin Decoction Combined with Docetaxel on Advanced Ovarian Cancer and the Effect on the Levels of Serum Markers VEGF, HE4, and CA125" was retracted in 2023. Reasons: signs of a paper mill; suspected computer-generated content; unreliable results or conclusions; lack of ethics approval or compliance.

## Data Availability

The data to support the findings of this study are available on reasonable request from the corresponding author.
